# LncRNA HAND2-AS1 inhibits non-small cell lung cancer migration, invasion and maintains cell stemness through the interactions with TGF-β1

**DOI:** 10.1042/BSR20181525

**Published:** 2019-01-11

**Authors:** Feng Miao, Ji Chen, Meng Shi, Yang Song, Zhiming Chen, Liewen Pang

**Affiliations:** Department of Thoracic Surgery, Huashan Hospital, Fudan University, Shanghai 200040, P.R. China

**Keywords:** invasion, lncRNA HAND2-AS1, migration, non-small cell lung cancer, TGF-β1

## Abstract

LncRNA HAND2-AS1 is characterized as a tumor suppressor involved in several types of malignancies, but its role in non-small cell lung cancer (NSCLC) is unknown. Our study was carried out to investigate the involvement of lncRNA HAND2-AS1 in NSCLC. In our study, we observed that levels of HAND2-AS1 were lower in tumor tissues than that in adjacent healthy tissues. Compared with healthy controls, plasma levels of HAND2-AS1 were lower, while levels of transforming growth factor β (TGF-β) were higher in NSCLC patients. A significant negative correlation between plasma levels of HAND2-AS1 and TGF-β1 was found in NSCLC patients but not in healthy controls. LncRNA HAND2-AS1 overexpression inhibits, while exogenous TGF-β1 treatment promotes cell migration and invasion ability and cancer cell stemness. Cancer cells with lncRNA HAND2-AS1 overexpression showed down-regulated TGF-β1, while TGF-β1 treatment showed no significant effects on lncRNA HAND2-AS1 expression. TGF-β1 attenuated the inhibitory effects of lncRNA HAND2-AS1 overexpression on cell migration, invasion and stemness. We concluded that lncRNA HAND2-AS1 may regulate the migration, invasion and stemness of NSCLC cells through interactions with TGF-β1.

## Introduction

Tumor metastasis, which is mediated by cancer cell invasion and migration, is the key step of cancer development. Therefore, how to predict and prevent cancer metastasis is a major task in cancer treatment and major cause of deaths among cancer patients [1–3]. As the major type of lung cancer, non-small cell lung cancer (NSCLC) is one of the most frequently diagnosed malignancies with unacceptable high mortality rate [4]. With the efforts have been made on the treatment of NSCLC, survival of patients at early stages has been improved significantly over past several decades [5]. However, once cancer metastasis occurs, prognosis will be extremely poor [6].

Transforming growth factor β (TGF-β) signaling pathway is a well-characterized pathway involved in cancer biology [7]. TGF-β signaling plays different roles in different stages of cancer development. At the initiation of tumor formation, TGF-β inhibits tumor cell proliferation to play a role as tumor suppressor [8]. In contrast, TGF-β promotes tumor metastasis by mediating epithelial–mesenchymal transition at late stages [9]. In NSCLC, inhibiting TGF-β signaling is considered as a promising target for cancer treatment [10]. A growing body of literatures has revealed that TGF-β signaling participates in cancer development and inhibits through the interactions not only with proteins but also with non-coding RNAs, such as lncRNAs [11]. LncRNA HAND2-AS1 is a well-characterized tumor suppressor in several types of malignancies [12–14]. In the present study, we showed that lncRNA HAND2-AS1 may also serve as a tumor suppressor in NSCLC through the inhibition of TGF-β1.

## Materials and methods

### Human tissues and cell lines

NCI-H1581 [H1581] and NCI-H1993 [H1993] human NSCLC cell lines were provided by American Type Culture Collection (ATCC, Manassas, VA, U.S.A.). Cells were cultivated in ATCC-formulated RPMI-1640 medium containing 10% fetal bovine serum (FBS, ATCC 30-2020) under normal conditions (37°C, 5% CO_2_).

Tumor tissues and adjacent healthy tissues were obtained from 72 NSCLC patients who were admitted by Huashan Hospital from May 2016 to May 2018. Inclusion criteria: (1) patients diagnosed as NSCLC at stage I and II through pathological examinations; (2) patients and their families understood the whole experimental protocol and signed informed consent. Exclusion criteria: (1) patients who were suffering from other diseases; (2) patients who were treated within 100 days before admission. Plasma was derived from blood extracted from the 72 NSCLC patients (patient group) and 54 healthy volunteers (control group). The 54 healthy volunteers received systemic physiological examinations in Huashan Hospital during the same time period. Patient group was composed of 40 males and 32 females, and age ranged from 36 to 65 years, with a mean age of 50.3 ± 5.1 years. Control group was composed of 30 males and 24 females, and age ranged from 34 to 66 years, with a mean age of 49.6 ± 5.5 years. Those two groups have similar age and gender distributions. Ethics committee of Huashan Hospital approved this study, all participants signed informed consent. Experiments using human materials were carried out in accordance with the World Medical Association Declaration of Helsinki (Ethics approval ID: 20151216).

### Enzyme-linked immunosorbent assay

Plasma levels of TGF-β1 were measured using a kit provided by Human TGF-β1 Quantikine ELISA Kit (DB100B, R&D Systems). TGF-β1 levels were normalized to ng/ml.

### Real-time quantitative PCR (qRT-PCR)

Monarch® Total RNA Miniprep Kit (NEB) was used to extract total RNA. Total RNA samples were subjected to reverse transcription using High-Capacity cDNA Reverse Transcription Kit (Thermo Fisher Scientific). Luna® Universal One-Step RT-qPCR Kit (NEB) was used to prepare all PCR reaction systems. Sequences of primers used in PCR reactions were: 5′-GGGTGTTTACGTAGACCAGAACC-3′ (forward) and 5′-CTTCCAAAAGCCTTCTGCCTTAG-3′ (reverse) for human lncRNA HAND2-AS1; 5′- GACCTCTATGCCAACACAGT3′ (forward) and 5′- AGTACTTGCGCTCAGGAGGA3′ (reverse) for β-actin. PCR reactions were perfromed according to following conditions: 95°C for 50 s, followed by 40 cycles of 95°C for 12 s and 57.5°C for 25 s. All *C*_t_ values were processed using 2^−ΔΔ*C*^_t_ method.

### Cell transfection

LncRNA HAND2-AS1 expression vectors were designed and synthesized by GenePharma (Shanghai, China). Cells were cultivated overnight to reach 80–90% confluence. Lipofectamine 2000 reagent (11668-019, Invitrogen, Carlsbad, U.S.A.) was used to transfect 10 nM vectors into cells. Cells without transfection were control cells. Cells transfected with empty vectors were negative control cells. Expression of lncRNA HAND2-AS1 was detected by qRT-PCR and overexpression rate above 200% was achieved before subsequent experiments (data not shown).

### Transwell migration and invasion assay

After transfection, cell suspensions (4 × 10^4^ cells/ml) were prepared using serum-free RPMI-1640 medium. Cells were transferred to the upper chamber with 0.1 ml of cell suspension for each well, while the lower chamber was filled with RPMI-1640 medium containing 20% FBS. After 24 h, 0.5% crystal violet (Sigma-Aldrich, U.S.A.) staining was performed at 25°C for 20 min. Invasion and migration assays were performed in the same way except that the upper chamber was pre-coated with Matrigel (356234, Millipore, U.S.A.) before invasion assay.

### Flow cytometry

Cells were harvested by trypsinization and were incubated with CD133-PE or IgG1-PE antibody (130-093-193, Meltenyi Biotec, Germany) for 15 min at 4°C. After that, cells were centrifuged and resuspended in PBS. FACS Aria system (BD Immunocytometry Systems, San Jose, CA, U.S.A.) was used to detect signals and signals were processed using Cell Quest software (Becton Dickinson Ltd).

### Western blotting

Total Protein Extraction Kit (2140, Merck Millipore) was used to extract total protein from *in vitro* cultured cells. Electrophoresis was performed using 12% SDS-PAGE gel. Western blot was performed using conventional method. Primary antibodies used in Western blot were rabbit anti-human TGF-β1 (ab9758, 1:1200; Abcam), rabbit anti-human p-Smad2/3 (ab63399, 1:1200; Abcam) and rabbit anti-human GAPDH (ab9485, 1: 1400, Abcam). Secondary antibody was goat anti-rabbit IgG-HRP secondary antibody (1:1000, MBS435036, MyBioSource). Signals were developed using ECL (Sigma-Aldrich, U.S.A.). Image J v.1.46 software was used for data normalization.

### Statistical analysis

All experiments were performed in triplicate manner and data were recorded as mean ± standard deviation. Comparisons between two groups were performed by Student’s *t* test. Comparisons among multiple groups were performed by one-way ANOVA followed by Tukey test. Correlation analyses were performed by Pearson correlation coefficient. ROC curve analysis was used for diagnostic analysis. *P*<0.05 was considered to be statistically significant.

## Results

### Expression of lncRNA HAND2-AS1 was altered in NSCLC and was negatively correlated with TGF-β1

Compared with adjacent healthy tissues, qRT-PCR results showed that expression levels of lncRNA HAND2-AS1 were significantly reduced in tumor tissues (Figure 1, *P*<0.05). Therefore, down-regulation of lncRNA HAND2-AS1 is very likely involved in NSCLC. In addition, compared with healthy volunteers, plasma levels of lncRNA HAND2-AS1 were significantly reduced in patients with NSCLC (Figure 2A, *P*<0.05). ROC curve analysis was performed with NSCLC patients as true positive cases and healthy volunteers as true negative cases, results showed that the area under the curve was 0.8695, with standard error of 0.03023 and 95% confidence interval of 0.8102–0.9287 (*P*<0.0001). ELISA results revealed significantly up-regulated plasma levels of TGF-β1 in NSCLC patients than in healthy controls (Figure 3A, *P*<0.05). Pearson correlation analysis showed that plasma levels of lncRNA HAND2-AS1 and TGF-β1 were negatively correlated in NSCLC patients (Figure 3B). However, the correlation between lncRNA HAND2-AS1 and TGF-β1 was not significant in healthy controls (Figure 3C).

**Figure 1:** Altered expression of lncRNA HAND2-AS1 was observed in tumor tissues compared with adjacent healthy tissues QRT-PCR results showed that expression levels of lncRNA HAND2-AS1 were significantly reduced in tumor tissues than in adjacent healthy tissues (*P<0.05).

**Figure 2:** Down-regulation of lncRNA HAND2-AS1 distinguished NSCLC patients from healthy controls QRT-PCR results showed that plasma levels of lncRNA HAND2-AS1 were significantly lower in patients with NSCLC than in healthy controls (**A**) (*P<0.05), and down-regulation of lncRNA HAND2-AS1 distinguished NSCLC patients from healthy controls (**B**).

**Figure 3:** Plasma TGF-β1 was up-regulated in NSCLC patients and was negatively correlated with lncRNA HAND2-AS1 ELISA data showed that plasma levels of TGF-β1 were significantly up-regulated in NSCLC patients than in healthy controls (**A**) (*P<0.05). Pearson’s correlation coefficient showed that plasma levels of lncRNA HAND2-AS1 and TGF-β1 were negatively correlated in NSCLC patients (**B**) but not in healthy controls (**C**).

### LncRNA HAND2-AS1 and TGF-β1 play opposite roles in the migration, invasion and stemness of cells of NSCLC cell lines H1581 and H1993

Transwell migration and invasion assay results showed that, compared with control cells (C) and negative control cells (NC), overexpression of lncRNA HAND2-AS1 significantly inhibited, while treatment with exogenous TGF-β1 at a dose of 10 ng/ ml (Sigma-Aldrich) significantly promoted the migration (Figure 4A, *P*<0.05) and invasion (Figure 4B, *P*<0.05) of cells of NSCLC cell lines H1581 and H1993. In addition, exogenous TGF-β1 treatment partially reversed the inhibitory effects of overexpression of lncRNA HAND2-AS1 on cancer cell migration (Figure 4A, *P*<0.05) and invasion (Figure 4B, *P*<0.05). Flow cytometric analysis results revealed that, compared with control cells (C) and negative control cells (NC), overexpression of lncRNA HAND2-AS1 significantly reduced, while treatment with exogenous TGF-β1 at doses of 10 ng/ml significantly increased the percentage of CD133+ cells of both H1581 and H1993 cell lines (Figure 5, *P*<0.05). In addition, compared with cells with lncRNA HAND2-AS1 overexpression alone, cells with both lncRNA HAND2-AS1 overexpression and exogenous TGF-β1 treatment showed significantly increased percentage of CD133+ cells (Figure 5, *P*<0.05).

**Figure 4:** LncRNA HAND2-AS1 and TGF-β1 play opposite roles in the migration and invasion of cells of NSCLC cell lines H1581 and H1993 Overexpression of lncRNA HAND2-AS1 significantly inhibited, while treatment with exogenous TGF-β1 at a dose of 10 ng/ ml (Sigma-Aldrich) significantly promoted the migration (**A**) and invasion (**B**) of cells of NSCLC cell lines H1581 and H1993. Exogenous TGF-β1 treatment significantly attenuated the inhibitory effects of overexpression of lncRNA HAND2-AS1 on cancer cell migration and invasion (*P<0.05).

**Figure 5:** LncRNA HAND2-AS1 and TGF-β1 play opposite roles in the stemness of cells of NSCLC cell lines H1581 and H1993 Overexpression of lncRNA HAND2-AS1 significantly reduced, while treatment with exogenous TGF-β1 at doses of 10 ng/ml significantly increased the percentage of CD133+ cells of both H1581 and H1993 cell lines. In addition, TGF-β1 treatment significantly attenuated the effects of lncRNA HAND2-AS1 overexpression on cell stemness (*P<0.05).

### LncRNA HAND2-AS1 regulates TGF-β1 expression in cells of NSCLC cell lines H1581 and H1993

Compared with control cells (C) and negative control cells (NC), overexpression of lncRNA HAND2-AS1 led to significant inhibited expression of TGF-β1 and reduced level of p-Smad2/3 in cells of both H1581 and H1993 cell lines (Figure 6A, *P*<0.05). In contrast, treatment with exogenous TGF-β1 at a doses of 10, 20 and 40 ng/ml showed no significant effects on lncRNA HAND2-AS1 expression in cells of both cell lines (Figure 6B).

**Figure 6:** LncRNA HAND2-AS1 regulates TGF-β1 expression in cells of NSCLC cell lines H1581 and H1993 Overexpression of lncRNA HAND2-AS1 led to significant inhibited expression of TGF-β1 and reduced level of p-Smad2/3 in cells of both H1581 and H1993 cell lines (**A**), while treatment with exogenous TGF-β1 at doses of 10, 20 and 40 ng/ml showed no significant effects on lncRNA HAND2-AS1 expression (**B**) (*P<0.05).

## Discussion

The tumor suppression role of lncRNA HAND2-AS1 has been well-characterized in several types of malignancies including osteosarcoma [12], colorectal cancer [13] and endometrioid endometrial carcinoma [14]. However, the involvement of lncRNA HAND2-AS1 in lung cancer is unknown. The main finding of our study is that lncRNA HAND2-AS1 is also likely a tumor suppressor in NSCLC, which is the major subtype of lung cancer. The tumor suppression function of lncRNA HAND2-AS1 is likely achieved through the inhibition of TGF-β signaling.

Cancer diagnosis at early stages is conductive for the survival of cancer patients. Although the involvement of lncRNA HAND2-AS1 in several types of cancers has already been reported [12–14], its potentials for cancer diagnosis is unknown. Our study found significantly inhibited expression of lncRNA HAND2-AS1 in tumor tissues than in adjacent healthy tissues of NSCLC patients. ROC curve analysis revealed that down-regulation of plasma lncRNA HAND2-AS1 distinguished NSCLC patients from healthy controls. It is worth to note that all the patients included in the present study is at stage I or II, which were early stages of cancer development and before the occurrence of cancer metastasis. *In vitro* cell experiments showed that lncRNA HAND2-AS1 overexpression inhibited cancer cell migration and invasion. Therefore, lncRNA HAND2-AS1 may be used to assist early diagnosis of NSCLC and lncRNA HAND2-AS1 overexpression may serve as a promising target for NSCLC treatment.

The activation of TGF-β has been observed in development of different types of cancers including NSCLC [15]. Consistently, our study also observed significantly up-regulated plasma TGF-β1 in NSCLC cancer patients than in healthy controls. Besides cancer growth and metastasis, TGF-β signaling also participates in the regulation of cancer stemness [16], which is also a mediator of cancer metastasis [17]. Our study showed that exogenous TGF-β1 promoted migration, invasion and stemness of NSCLC cells. It is known that TGF-β can be regulated by lncRNAs in cancer biology [18,19]. Interestingly, our study identified lncRNA HAND2-AS1 as a potential upstream inhibitor of TGF-β1 in the regulation of migration, invasion and stemness of NSCLC cells. Further studies on the phosphorylation of Smad2/3 revealed that lncRNA HAND2-AS1 inhibits TGF-β/Smad pathway. However, the lack of significant correlation between lncRNA HAND2-AS1 and TGF-β1 revealed that the role of lncRNA HAND2-AS1 in regulating the activation of TGF-β/Smad pathway is likely indirect. It is also worth to note that lncRNA HAND2-AS1 may interact with multiple functional molecules in the regulation of migration, invasion and stemness of NSCLC cells due to the fact that exogenous TGF-β1 only partially not totally reversed the inhibitory effects of lncRNA HAND2-AS1 overexpression on migration, invasion and stemness of NSCLC cells.

Interesting, in a recently study, Wang et al. [20] reported that lncRNA ANCR inhibited the migration and invasion of cancer cells of NSCLC also through the interactions with TGF-β. Therefore, TGF-β may participate in the same pathological processes through the interactions with multiple lncRNAs. It is possible that any lncRNA transfections can induce the altered expression of TGF-β pathway and future studies should investigate this possibility.

In conclusion, lncRNA HAND2-AS1 is down-regulated in NSCLC. LncRNA HAND2-AS1 overexpression inhibited migration, invasion and stemness of NSCLC cells by down-regulating TGF-β1.

## Abbreviations

NSCLC: non-small cell lung cancer
TGFβ: transforming growth factor β

## References

[1] SathiakumarN., DelzellE., MorriseyM.A., FalksonC., YongM., ChiaV. (2011) Mortality following bone metastasis and skeletal-related events among men with prostate cancer: a population-based analysis of US Medicare beneficiaries, 1999-2006. Prostate Cancer Prostatic Dis. 14, 177–183 10.1038/pcan.2011.7 21403668

[2] ReckM., PopatS., ReinmuthN., De RuysscherD., KerrK.M., PetersS. (2014) Metastatic non-small-cell lung cancer (NSCLC): ESMO Clinical Practice Guidelines for diagnosis, treatment and follow-up. Ann. Oncol. 25, iii27–iii39 10.1093/annonc/mdu199 25115305

[3] MinnA.J., GuptaG.P., SiegelP.M., BosP.D., ShuW., GiriD.D. (2005) Genes that mediate breast cancer metastasis to lung. Nature 436, 518–524 10.1038/nature03799 16049480PMC1283098

[4] EttingerD.S., AkerleyW., BorghaeiH. (2012) Non-small cell lung cancer. J. Natl. Compr. Canc. Netw. 10, 1236–1271 10.6004/jnccn.2012.0130 23054877

[5] CrinoL., WederW., van MeerbeeckJ., FelipE. and GroupE.G.W. (2010) Early stage and locally advanced (non-metastatic) non-small-cell lung cancer: ESMO Clinical Practice Guidelines for diagnosis, treatment and follow-up. Ann. Oncol. 21, v103–v115 10.1093/annonc/mdq207 20555058

[6] NovelloS., BarlesiF., CalifanoR., CuferT., EkmanS., LevraM.G. (2016) Metastatic non-small-cell lung cancer: ESMO Clinical Practice Guidelines for diagnosis, treatment and follow-up. Ann. Oncol. 27, v1–v27 10.1093/annonc/mdw326 27664245

[7] DerynckR., AkhurstR.J. and BalmainA. (2001) TGF-beta signaling in tumor suppression and cancer progression. Nat. Genet. 29, 117–129 10.1038/ng1001-117 11586292

[8] AkhurstR.J. and DerynckR. (2001) TGF-beta signaling in cancer–a double-edged sword. Trends Cell Biol. 11, S44–S51 1168444210.1016/s0962-8924(01)02130-4

[9] CaoM., SeikeM., SoenoC., MizutaniH., KitamuraK., MinegishiY. (2012) MiR-23a regulates TGF-beta-induced epithelial-mesenchymal transition by targeting E-cadherin in lung cancer cells. Int. J. Oncol. 41, 869–875 10.3892/ijo.2012.1535 22752005PMC3582905

[10] YuanJ.H., YangF., WangF. (2014) A long noncoding RNA activated by TGF-beta promotes the invasion-metastasis cascade in hepatocellular carcinoma. Cancer Cell 25, 666–681 10.1016/j.ccr.2014.03.010 24768205

[11] SaitoT., KurashigeJ., NambaraS. (2015) A long non-coding RNA activated by transforming growth factor-beta is an independent prognostic marker of gastric cancer. Ann. Surg. Oncol. 22, S915–S922 10.1245/s10434-015-4554-8 25986864

[12] KangY., ZhuX., XuY., TangQ., HuangZ., ZhaoZ. (2018) Energy stress-induced lncRNA HAND2-AS1 represses HIF1alpha-mediated energy metabolism and inhibits osteosarcoma progression. Am. J. Cancer Res. 8, 526–537 29637006PMC5883101

[13] ZhouJ., LinJ., ZhangH., ZhuF. and XieR. (2018) LncRNA HAND2-AS1 sponging miR-1275 suppresses colorectal cancer progression by upregulating KLF14. Biochem. Biophys. Res. Commun. 503, 1848–18533007867710.1016/j.bbrc.2018.07.125

[14] YangX., WangC.C., LeeW.Y.W., TrovikJ., ChungT.K.H. and KwongJ. (2018) Long non-coding RNA HAND2-AS1 inhibits invasion and metastasis in endometrioid endometrial carcinoma through inactivating neuromedin U. Cancer Lett. 413, 23–34 10.1016/j.canlet.2017.10.028 29107108

[15] YangH., WangL., ZhaoJ., ChenY., LeiZ., LiuX. (2015) TGF-beta-activated SMAD3/4 complex transcriptionally upregulates N-cadherin expression in non-small cell lung cancer. Lung Cancer 87, 249–257 10.1016/j.lungcan.2014.12.015 25595426

[16] BellomoC., CajaL. and MoustakasA. (2016) Transforming growth factor beta as regulator of cancer stemness and metastasis. Br. J. Cancer 115, 761–769 10.1038/bjc.2016.255 27537386PMC5046208

[17] MonteiroJ. and FoddeR. (2010) Cancer stemness and metastasis: therapeutic consequences and perspectives. Eur. J. Cancer 46, 1198–1203 10.1016/j.ejca.2010.02.030 20303259

[18] ZhaoB., LuY.L., YangY., HuL.B., BaiY., LiR.Q. (2018) Overexpression of lncRNA ANRIL promoted the proliferation and migration of prostate cancer cells via regulating let-7a/TGF-beta1/ Smad signaling pathway. Cancer Biomark. 21, 613–620 10.3233/CBM-170683 29278879PMC5859458

[19] WangX., WangG., ZhangL., CongJ., HouJ. and LiuC. (2018) LncRNA PVT1 promotes the growth of HPV positive and negative cervical squamous cell carcinoma by inhibiting TGF-beta1. Cancer Cell Int. 18, 70 10.1186/s12935-018-0567-2 29760583PMC5941374

[20] WangS., LanF. and XiaY. (2018) lncRA ANCR inhibits non-small cell lung cancer cell migration and invasion by inactivating TGF-β pathway. 24, 6002–600910.12659/MSM.911492PMC612641530154397

